RETRACTED

# Identifying COVID-19-Specific Transcriptomic Biomarkers with Machine Learning Methods

**DOI:** 10.1155/2021/9939134

**Published:** 2021-07-06

**Authors:** Lei Chen, Zhandong Li, Tao Zeng, Yu-Hang Zhang, KaiYan Feng, Tao Huang, Yu-Dong Cai

**Affiliations:** ^1^School of Life Sciences, Shanghai University, shanghai 200444, China; ^2^College of Information Engineering, Shanghai Maritime University, shanghai 201306, China; ^3^College of Food Engineering, Jilin Engineering Normal University, Changchun 130052, China; ^4^Bio-Med Big Data Center, CAS Key Laboratory of Computational Biology, Shanghai Institute of Nutrition and Health, University of Chinese Academy of Sciences, Chinese Academy of Sciences, shanghai 200031, China; ^5^Channing Division of Network Medicine, Brigham and Women's Hospital, Harvard Medical School, Boston, MA, USA; ^6^Department of Computer Science, Guangdong AIB Polytechnic College, Guangzhou 510507, China; ^7^CAS Key Laboratory of Tissue Microenvironment and Tumor, Shanghai Institute of Nutrition and Health, University of Chinese Academy of Sciences, Chinese Academy of Sciences, Shanghai 200031, China

## Abstract

COVID-19, a severe respiratory disease caused by a new type of coronavirus SARS-CoV-2, has been spreading all over the world. Patients infected with SARS-CoV-2 may have no pathogenic symptoms, i.e., presymptomatic patients and asymptomatic patients. Both patients could further spread the virus to other susceptible people, thereby making the control of COVID-19 difficult. The two major challenges for COVID-19 diagnosis at present are as follows: (1) patients could share similar symptoms with other respiratory infections, and (2) patients may not have any symptoms but could still spread the virus. Therefore, new biomarkers at different omics levels are required for the large-scale screening and diagnosis of COVID-19. Although some initial analyses could identify a group of candidate gene biomarkers for COVID-19, the previous work still could not identify biomarkers capable for clinical use in COVID-19, which requires disease-specific diagnosis compared with other multiple infectious diseases. As an extension of the previous study, optimized machine learning models were applied in the present study to identify some specific qualitative host biomarkers associated with COVID-19 infection on the basis of a publicly released transcriptomic dataset, which included healthy controls and patients with bacterial infection, influenza, COVID-19, and other kinds of coronavirus. This dataset was first analysed by Boruta, Max-Relevance and Min-Redundancy feature selection methods one by one, resulting in a feature list. This list was fed into the incremental feature selection method, incorporating one of the classification algorithms to extract essential biomarkers and build efficient classifiers and classification rules. The capacity of these findings to distinguish COVID-19 with other similar respiratory infectious diseases at the transcriptomic level was also validated, which may improve the efficacy and accuracy of COVID-19 diagnosis.

RETRACTED

## 1. Introduction

COVID-19 is recognized as starting from the end of 2019. It is a severe respiratory disease caused by a new type of coronavirus SARS-CoV-2 and has been spreading all over the world [1–3]. By the end of January 2021, approximately 100 million cases and 2 million deaths have been reported worldwide [4], making COVID-19 one of the most widespread and deadly infectious diseases in human history. In the US alone, more than 26 million cases were reported [4]. Different from other severe diseases, COVID-19 hardly has typical symptoms that could be used for diagnosis. A wide range of disease-associated symptoms, such as respiratory or systematic, were reported to be associated with COVID-19, including fever, cough, headache, diarrhea, and muscle or body aches [5, 6]. Moreover, patients infected with SARS-CoV-2 may have no pathogenic symptoms, i.e., presymptomatic patients and asymptomatic patients. In the early stage (first 2 days) of SARS-CoV-2 infection, patients may not have any COVID-19 associated symptoms, and they could be clustered as presymptomatic patients [7]. However, some patients may never have any symptoms but still have been infected by SARS-CoV-2, and they could be defined as asymptomatic patients. Both types of patients could further spread the virus to other susceptible people, thereby making the control of the COVID-19 pandemic difficult [8].

The two major challenges for COVID-19 diagnosis at present are as follows: (1) patients could share similar symptoms with other respiratory infections, and (2) patients may not have any symptoms but could still spread the virus. Therefore, identifying new biomarkers at different omics levels (genomic, transcriptomic, or proteomic levels) may be helpful for large-scale screening and diagnosis of COVID-19. Genomic analyses on COVID-19 mainly focused on the genomics of the virus and not the host by identifying the typical sequence of the ORF1ab, spike, ORF3a, envelope, membrane, and nucleocapsid of SARS-CoV-2 [9]. Meanwhile, many transcriptomic and proteomic analyses focused on the host, especially on the host–virus interaction-associated alterations in the host system. For example, in April 2020, a systematic study (GSE150728) on the expression pattern of immune-associated genes in lung tissue or related human lung cells during the infection of SARS-CoV-2 was presented, revealing that the selective death of type II pneumocytes caused by abnormal immune responses caused high morbidity and mortality in COVID-19 cases [10]. However, despite the encouraging results presented, this study has two obvious shortcomings: (1) the major findings were based on in vitro-cultured cell lines and only two patients each group were enrolled, and (2) only immune-associated genes were taken into consideration. As for other transcriptomic analyses, only single-cell subgroups, such as human lung cell lines [10], cardiomyocyte cells [11], and human bronchial organoids [12], have been analysed and discussed, and systematic transcriptomic analyses on lung tissue are lacking.

RETRACTED

Although some initial analyses on such transcriptomic datasets could identify a group of candidate gene biomarkers, such as IFI6, TIMP1, and LGR6, for COVID-19 in the previous study [13], the dataset used did not contain normal controls and only divided patients into three rough groups: patients with COVID-19, those with other viral infections, and those without viral infections. Thus, the previous work could not fully identify biomarkers capable for clinical use in COVID-19, which requires disease-specific diagnosis compared with other multiple infectious diseases. As an extension of the previous study, a recent dataset released on the Gene Expression Omnibus (GEO) database (GSE161731) [14] was introduced for further analyses. These blood sample transcriptomic data of 195 subjects include 19 healthy controls and 23, 17, 77, and 59 patients with bacterial infection, influenza, COVID-19, and other kinds of coronavirus, respectively. The new dataset could be used to screen out potential transcriptomic biomarkers from the comprehensive lung tissue, and a comparison between COVID-19 and other infectious respiratory diseases could further help identify disease-specific biomarkers to distinguish COVID-19 from other similar diseases.

In this study, on the basis of the publicly released dataset, optimized machine learning models were applied to identify some specific qualitative host biomarkers associated with COVID-19 infection. Two powerful feature selection methods (Boruta [15] and Max-Relevance and Min-Redundancy (mRMR) [16]), were applied on this dataset one by one. A feature list was generated, which was further fed into the incremental feature selection (IFS) method [17]. Four classic classification algorithms were tried in the IFS method. As a result, we accessed some essential biomarkers, efficient classifiers, and classification rules. The capacity of these findings to distinguish COVID-19 with other similar respiratory infectious diseases at the transcriptomic level was validated, which could improve the efficacy and accuracy of COVID-19 diagnosis.

RETRACTED

## 2. Materials and Methods

### 2.1. Data

The blood expression profiles of 15,379 genes in acute respiratory infection samples were downloaded from the GEO database under accession number GSE161731 [14]. A total of 195 samples with demographic information were included as follows: 19 healthy controls, 23 patients with bacterial pneumonia, 17 patients with influenza, 59 patients with seasonal coronavirus, and 77 patients with SARS-CoV-2 infection. The 15,379 genes are listed in Table S1. The processed transcript-per-million expression data were used for further analysis.

### 2.2. Boruta Feature Filtering

The investigated dataset involved lots of features/genes. Evidently, some are relevant to acute respiratory infection, whereas others are not. To extract the relevant features, the Boruta [15] method was employed.

Boruta is a random forest- (RF-) based feature select method. Given a dataset, a shuffled feature is added for each original feature. A RF classifier is built on a dataset with original and added features. According to the performance of RF, calculate the *Z* score of all features and find the maximum *Z* score among shuffled features (MZSA). Determine the original features as “important” if their *Z* scores are significantly higher than MZSA; whereas when *Z* scores of some features are signicantly lower than MZSA, they are labelled as “unimportant.” The above procedures are executed several times until all original features are labelled as “important” or “unimportant,” or the times of RF runs have reached a predefined number.

In this study, we adopted the program of Boruta retrieved from https://github.com/scikit-learn-contrib/boruta_py. It was run with its default parameters.

### 2.3. Max-Relevance and Min-Redundancy (mRMR) Feature Selection

mRMR [16] is a mutual information- (MI-) based feature selection approach to evaluate the importance of features. This method has wide applications in tackling several biological and medical problems [13, 18–23]. For variables *x* and *y*, their MI can be calculated by

(1) $$\begin{array}{c} I\left(x,y\right)=\iint p\left(x,y\right)\log\frac{p\left(x,y\right)}{p\left(x\right)p\left(y\right)}dxdy, \end{array}$$

where *p*(*x*) denotes the marginal probabilistic density of *x*, *p*(*x*, *y*) represents the joint probabilistic density of *x* and *y*, respectively. A high MI means two variables have high associations. For a feature, its importance is reflected by its rank in a feature list. To generate such list, a loop procedure is included in the mRMR method. Initially, this list is empty. A feature is selected in each round and appended to this list. Such feature is selected by the following manner. For each nonselected feature, calculate its relevance to class labels, which is defined as the MI of it and class labels, and its redundancies to already-selected features, which is defined as the average MI of it and already-selected features. The feature with maximum difference of above two values is selected. The loop procedure stops until all features are selected. For convenience, this list was called mRMR feature list in this study.

RETRACTED

In present study, the mRMR program downloaded from http://penglab.janelia.org/proj/mRMR/ was used. Such program was executed with its default parameters.

### 2.4. Incremental Feature Selection (IFS)

IFS is a widely used approach integrated with supervised classifier (e.g., SVM) to determine the optimal feature number for classification model construction [17]. On the basis of the mRMR feature list available from mRMR, IFS could produce step-wise feature subsets in a given step interval *s* (i.e., 1). For instance, the first feature subset has the top-ranked *s* features, and then the second feature subset has the top-ranked 2 × *s* features, and so on. For each candidate feature subset, a classifier could be built on the basis of the training sample data within such feature subset. In IFS, the optimal feature subset is obtained when a classifier could achieve the best performance measurement, evaluated by Matthew's correlation coefficient (MCC) [24], within 10-fold cross-validation [25] on such feature subset.

### 2.5. Candidate Classification Algorithms

The four classification algorithms were tried in the IFS method. Their brief descriptions are as follows.

#### 2.5.1. RF

RF is an assembly prediction model that uses average prediction [26], which predicts the class label of a test sample dependent on the consensus prediction results from a series of decision trees (DTs). It is widely used in bioinformatics researches [27–31].

#### 2.5.2. Support Vector Machine (SVM)

SVM [32–38] consists of several computational steps. First, it transforms the original data from a low-dimensional data space to a high-dimensional data space. It could also transform the original nonlinear data pattern to new linear data pattern [39, 40]. Second, it divides the data points in the high-dimensional data space by maximizing the space interval among data points from different classes/labels. Finally, it predicts the test sample's class label by judging which space interval this new data point belongs to. Here, the SVM model construction adopted the SMO in Weka.

RETRACTED

#### 2.5.3. *K*-Nearest Neighbor (kNN)

The computational steps of kNN [41] are as follows: first, it calculates the sample distance between a new sample and all training samples. Then, it ranks all training samples in accordance with these distance measurements. Next, it chooses the *K*-nearest training samples and estimates the class label distribution of these samples. Finally, it predicts the class label of new sample as the one with the largest distribution frequency. Here, the kNN model building adopted the Ibk in Weka.

#### 2.5.4. DT

As a rule-based white-box classification and regression model, DT [42, 43] generally applies IF-TEHN format to indicate each feature's role and weight in a model and corresponding rule, which thereby provides interpretative rules. Here, the DT model learning adopted the CART algorithm with the Gini index in the Scikit-learn package.

### 2.6. MCC

MCC [24] can evaluate the classification performance of different models. For the multiclass problem faced in this work, MCC could be calculated using the following formula:

(2) $$\begin{array}{c} \text{MCC}=\frac{\mathrm{cov}\left(X,Y\right)}{\sqrt{\mathrm{cov}\left(X,X\right)\mathrm{cov}\left(Y,Y\right)}}, \end{array}$$

where data matrix *X* has binary values representing the predicted sample classes, data matrix *Y* has binary values indicating the true sample classes, and cov(·, ·) calculates the two matrices' covariance. The value of MCC ranges from −1 to +1 [19], and it is equal to +1 when the classification model has the best performance.

## 3. Results

In this study, we applied several advanced computational methods to the blood expression profiles of acute respiratory infection samples. The whole procedures are illustrated in Figure 1. The detailed results are listed in this section.

### 3.1. Results of Boruta and mRMR Methods

Each acute respiratory infection sample was represented by the blood expression level of 15,379 genes, which are provided in Table S1. These features (genes) were first analysed by the Boruta method. 604 relevant features were extracted, which are listed in Table S2. Then, these features were evaluated by the mRMR method. A feature list, called mRMR feature list, was produced, which is also provided in Table S2.

### 3.2. Results of IFS Method

The mRMR feature list was fed into the IFS method, which incorporated one of four classification algorithms (RF, SVM, KNN, and DT). 604 feature subsets were constructed in the IFS method, each of which contained some top features in the mRMR feature list. On each feature subset, a classifier was built based on a given classification algorithm, which was further assessed by 10-fold cross-validation. The accuracy on each category, overall accuracy, and MCC were counted. The above measurements obtained by all classification algorithms and constructed feature subsets are available in Table S3. For an easy observation, a curve was plotted for each classification algorithm, in which MCC was set as the *Y*-axis and number of features was set as the *X*-axis. These four curves are shown in Figure 2. For SVM, the highest MCC was 0.917, which was obtained by using top 168 features. Thus, the SVM classifier with these features was deemed as the optimum SVM classifier. The overall accuracy of such classifier was 0.938 (Table 1). The accuracies on five categories yielded by such classifier are illustrated in Figure 3. Samples in three categories were all correctly predicted. These results indicated the excellent performance of the optimum SVM classifier.

RETRACTED

As for KNN and RF, the highest MCCs were 0.845 and 0.896 when the top 183 and 565, respectively, features were used. These MCCs were lower than that of the optimum SVM classifier. Likewise, the optimum KNN and RF classifiers were built with the corresponding top features. The overall accuracies of these two classifiers are listed in Table 1. They were also lower than that of the optimum SVM classifier. The accuracies on five categories yielded by these two classifiers were also generally lower than those of the optimum SVM classifier (see Figure 3).

In addition to the above-mentioned three black-box classification algorithms, we also employed a white-box classification algorithm, DT. The same procedure was done for this algorithm. The curve is shown in Figure 2. The highest MCC was 0.818 when top 511 features were adopted. Such MCC was lower than that of the optimum SVM/KNN/RF classifier. The overall accuracy was 0.867 (Table 1), also lower than that of the optimum SVM/KNN/RF classifier. Furthermore, the accuracies on five categories, as shown in Figure 3, were also generally lower than those of other three optimum classifiers. Although such DT classifier did not provide good performance, we can obtain more insights from such classifier, which would be listed in the following subsection.

### 3.3. Classification Rules

The best DT classifier adopted top 511 features. Thus, we used these 511 features to build a DT using all acute respiratory infection samples. 21 rules were extracted from this DT, which are listed in Table S4. Among these 21 rules, eight rules were for prediction of SARS-CoV-2 infection samples, which were most, followed by rules for seasonal coronavirus, influenza, healthy control, and bacterial pneumonia (see Figure 4). The discussion on these rules can be found in Discussion.

RETRACTED

### 3.4. Functional Enrichment Analyses

The optimum SVM classifier adopted top 168 features (genes). Using these selected COVID19 associated genes as gene of interest and all genes in analyses as gene background, we performed GO and KEGG enrichment analyses using DAVID website (https://david.ncifcrf.gov/). The FDR threshold for significant enriched results is set as 0.05. All the significant results are presented in Table 2.

## 4. Discussion

The top-ranked features (genes/transcripts) and rules were identified by applying these optimal machine learning models. According to recent publications [44–51], several identified top-ranked features and rule-involved features have been confirmed to be associated with the infection of a specific kind of pathogen, thus validating the efficacy and accuracy of the prediction in the current work. The detailed discussion can be found below.

### 4.1. Transcripts Associated with Disease-Specific Diagnosis of Different Pathogens

The first identified gene in the prediction list is ***RPL6***. Together with some other ribosomal proteins, such as ***RPL3*** and ***RPS20***, *RPL6* has already been reported to have differential expression patterns under specific physical and pathological conditions [52, 53]. Early in 2006, ribosomal proteins have been shown to be associated with lung bacterial infections caused by pneumococcal pneumonia in a mouse model [44]. As for influenza virus infections, in 2015, another independent study [45] at transcriptomic level has identified a group of ribosomal proteins, including *RPL6*, *RPL15*, *RPL17*, and *RPL22*, to have differential expression levels during influenza infections. As for coronavirus, including SARS-CoV-2, in 2020, a study [54] on the interactions between viral envelope protein and host cells confirmed that papain-like proteases, which are quite conserved in the coronavirus family, interact with the host ribosomal proteins. Therefore, ribosomal proteins, such as *RPL6*, *RPL3*, and *RPS20*, have differential expression levels during bacterial infection, influenza, and coronavirus infections, including COVID, thus making such transcripts potential biomarkers to distinguish patients with viral infections and normal controls.

The next identified gene is ***ZNF496***, an effective DNA-binding transcription factor in the lung under physical and pathological conditions [55]. With few validated reports on its associations with infections, it has only been shown to be associated with SARS-CoV-2 in a recent transcriptional regulatory network study [46] and identified as a potential therapeutic target, implying its potential significance for COVID-19 [46]. Therefore, such gene may also be a potential biomarker distinguishing patients with COVID-19 from others.

RETRACTED

***DYNLRB1***, as another predicted biomarker candidate, has previously been reported to be associated with linking dynein to cargos and regulatory adapters for dynein functions [56]. Early in 2011, *DYNLRB1* has been confirmed to be associated with multiple viral infections in lung, including influenza virus but not coronavirus, in mouse models [47]. However, no direct evidence has shown that such gene is associated with bacterial or coronavirus infections (including COVID-19), indicating it may be a potential biomarker for influenza virus infection, which is also in agreement with the prediction.

***TRBV20-1*** is a transcript of the variable domain of T cell receptor, which participates in the antigen recognition and varies for different potential antigens, such as those from different pathogens, including influenza, bacteria, or coronavirus [48, 49]. Although gene *TRBV20-1* does not have tissue specificity, considering that T cell-mediated immune responses have shown to be associated with COVID infections and the predicted gene *TRBV20-1* has been confirmed to be expressed in lung, it is reasonable to speculate that *TRBV20-1* may participate in the COVID-mediated lung infections.

Apart from another ribosomal protein associated transcript ***RPL36AL***, ***PHOSPHO1***, as a potential regulator for phosphatase activity and phosphocholine phosphatase activity regulations in cells, has been predicted to have differential expression levels during infection with different pathogens. Phosphatase activity has been shown to be essential for the infection of bacteria [57], influenza [58], and SARS-CoV-2 [50]. In particular, in the study associated with SARS-CoV-2, *PHOSPHO1* has also been shown to be associated with immunomodulatory effects of the host against such virus [50]. Therefore, *PHOSPHO1* may also be one of the potential biomarker candidates with disease-specific diagnosis capacity.

***TMEM165***, as a widely reported transmembrane protein expressed in fibroblasts, has also been predicted to be associated with bacterial infections in lungs. Different from the genes discussed above, *TMEM165* has been shown to be not associated with viral infections, including influenza or coronavirus infection. In 2019, researchers have shown that *TMEM165* is associated with bacterial infections in yeast [59]. Further, another study confirmed that such gene is effective in the lung and associated with chronic bacterial infection and inflammation [51], thus corresponding with the prediction in the present work.

### 4.2. Quantitative Rules Associated with Disease-Specific Diagnosis of Different Pathogens

Apart from the above qualitative analyses, quantitative analyses were performed to establish accurate rules for disease classification. Here, the top rules of each group were selected for follow-up detailed discussion.

RETRACTED

The first rule aims to identify patients with COVID-19 infection with decreased expression levels of ***SORT1***, ***RPL21P28***, ***SIDT2***, and ***TKT*** and a relatively high expression of **GZMB**. ***SORT1*** has been shown to be upregulated in almost all lung infections due to its specific relationships with neutrophil recruitment in lung tissues/surrounding vascular against pathogens, especially for bacterial infections [60–62]. By contrast, specifically, in COVID-19, a network based analyses has shown that such gene is associated with the infection of SARS-CoV-2 with a relatively low expression, corresponding with our predictions [63]. Similar decreased expression levels of *RPL21P28*, *SIDT2*, and *TKT* have also been validated in the transcriptomic analyses of COVID-19 host cells [64, 65]. Generally, *GZMB* has been widely reported to be expressed within cytotoxic CD8+ T cells. However, recent publications have also confirmed that in anti-virus CD4+ T cells, *GZMB* is also highly expressed which is detected using intracellular staining [66]. As specific for SARS-CoV-2 associated infections, in 2020, a specific single-cell transcriptomic analyses on SARS-CoV-2 host cells revealed that in reactive CD4+ T cells, ***GZMB*** turned out to be upregulated [67], corresponding with the prediction in the present study. Although based on our bulk analyses, we cannot confirm whether detected *GZMB* is derived from CD4+ or CD8+ T cells; however, as an SARS-CoV-2 viral infection-associated gene, the identification of such gene may also prove the validity of the prediction to a certain extent.

The next rule is aimed at identifying patients with other coronavirus infection with decreased expression levels of ***HK3***, ***CDKN1A***, ***HMGN3***, ***CACNA1l***, and ***ATP6V1D*** and an increased expression of ***SORT1***. As discussed above, *SORT1* has been shown to be associated with lung infections induced by multiple pathogens [60–62], including other coronavirus, thus explaining the high expression of such gene in this rule. *HK3*, which encodes the effective hexokinase 3 protein and participates in glucose metabolism pathways, has been predicted to be downregulated during coronavirus infection [68], including SARS-CoV-2 infection [69]. As for the remaining four genes, *CKDN1A* has been directly reported to be positively associated with coronavirus infection and related complications [70]. Although no direct evidence confirmed the relationship between coronavirus infection and *HMGN3*, *CACNA1l*, and *ATP6V1D*, all these genes have been shown to be associated with infection-associated inflammation responses [71, 72], indicating their potential capacity for the prediction of coronavirus infections.

RETRACTED

In rules associated with bacterial lung infections, the high expression levels of ***SORT1***, ***HK3***, and ***BAZ1A*** may be enough to identify patients with bacterial lung infections. As discussed above, a high expression of *SORT1* indicates the activation of neutrophil recruitment, which is quite common for bacterial infections [73] and different from COVID-19 infection. Meanwhile, *HK3* seems to be upregulated in lungs during bacterial infection, and such gene has been screened out as a host transcriptomic biomarker for the classification of bacteria and virus [74], thus corresponding with the prediction in the present work. Although no direct reports indicated the expression patterns of *BAZ1A* during bacterial infections, as mentioned above, neutrophil recruitment is quite common for bacterial infections.

With the involvement of effective biomarker candidates, such as ***SORT1***, ***HK3***, ***CDKN1A***, ***NLRC5***, and ***DACH1***, the next rule contributes to the identification of influenza virus infections. Similar with the previous rules, *SORT1*, *HK3*, and *CDKN1A* have been predicted to be associated with the identification of influenza virus infections. As discussed above, a high expression of *SORT1*, a downregulated *HK3*, and a high expression of *CDKN1A* are associated with viral infections [60–62, 68, 71, 72]. The upregulation of *NLRC5* and the activation of related pathways triggered by interactions between *NLRC5* and RIG-I initiate a robust antiviral response against influenza virus infection [75]. Therefore, a relatively increased expression of *NLRC5* during influenza virus infections is reasonable. As for *DACH1*, a recent comparable study [76] on COVID-19 infection, influenza virus infection, and normal controls revealed that after transcriptional regulation, the expression of *DACH1* was relatively increased in patients infected with influenza, thus validating the efficacy and accuracy of the newly presented computational methods.

Increased expression levels of ***RPL21P28*** and ***RTN1*** and a decreased expression of ***SORT1*** contribute to the rule for identifying healthy controls. The decreased expression of *SORT1* indicated no remarkable neutrophil recruitment, corresponding with the physical conditions of normal controls. *RPL21P28* has shown to be significantly differentially expressed in normal controls and tissues after infections, especially in human macrophages [77], which are generally activated during infections. Therefore, such gene could be summarized in this rule for the identification of normal controls. Similarly, *RTN1* has been shown to be associated with macrophage-mediated immune suppressants, different from the immune activators in the previously discussed rules [78], thereby validating the predictions on normal control.

RETRACTED

### 4.3. Functional Enrichment Analyses Using DAVID (DAVID Bioinformatics Resources 6.8)

Here, with the 168 selected COVID19 associated genes as gene of interest and all candidate genes as gene background, we performed functional enrichment analyses on GO terms and KEGG pathways using DAVID (Table 2) and selected the significant enriched results with FDR threshold as 0.05. According to the enriched results, multiple GO terms and KEGG pathways associated with RNA binding and replication via reverse transcription processes have been identified, meaning that selected genes are shown to be enriched in the RNA viral replication. Considering that COVID19 is a typical RNA virus, the enrichment results validated the reliability of the selected genes. Apart from that, we also identified multiple GO/KEGG terms associated with extracellular exosome/matrix. According to recent publications, extracellular microenvironment, especially for the vesicles outside the cells, is associated with the proliferation and spread of COVID-19 virus [79], validating our enrichment results.

All in all, the optimal blood-oriented features identified for the disease-specific diagnosis of COVID-19 and similar respiratory infectious pathogens have been validated. They are associated with their respective pathogens, and they even directly contribute to the pathogenesis according to recent publications. Therefore, the newly presented computational method in this study could be effective for the identification of COVID-19-associated biomarkers, and they could lay a solid foundation for further pathogenesis exploration on COVID-19-associated diseases.

## 5. Conclusion

In this study, a computational analysis was performed on an existing dataset of acute respiratory infection samples. The results included three parts. The first part was a set of genes/transcripts. They were highly related to one or more types of acute respiratory infection and can be latent biomarkers. The second part was the efficient classifiers, which can quickly identify the type of acute respiratory infection for a query sample. The third part was a set of classification rules, indicating different expression patterns on five types, giving more information to help us understand different types of acute respiratory infection.

RETRACTED

## Figures and Tables

**Figure 1:** Entire procedures to investigate the blood expression profiles of acute respiratory infection samples. The profiles are retrieved from Gene Expression Omnibus. They are first analysed by Boruta and mRMR methods, resulting in a feature list. Such list is fed into the incremental feature selection method to extract essential biomarker genes/transcripts, build efficient classifiers, and construct classification rules.

**Figure 2:** IFS curves with different classifiers on different numbers of gene features. The SVM provides the highest MCC of 0.917 when top 168 features are adopted.

**Figure 3:** Performance of the optimum classifiers with four different classification algorithms on five categories.

**Figure 4:** Pie chart to show the distribution of 21 classification rules on five categories.

**Table 1:** Performance of the optimum classifiers based on different classification algorithms.

Classification algorithm	Number of features	Overall accuracy	MCC
Decision tree	511	0.867	0.818
*K*-nearest neighbor	183	0.882	0.845
Support vector machine	168	0.938	0.917
Random forest	565	0.923	0.896

**Table 2:** Gene Ontology and KEGG pathway enrichment results.

Index	Term	Category
1	SRP-dependent cotranslational protein targeting to membrane	GOTERM_BP_DIRECT
2	Viral transcription	GOTERM_BP_DIRECT
3	Nuclear-transcribed mRNA catabolic process, nonsense-mediated decay	GOTERM_BP_DIRECT
4	Translational initiation	GOTERM_BP_DIRECT
5	Ribosome	KEGG_PATHWAY
6	Ribosome	GOTERM_CC_DIRECT
7	Translation	GOTERM_BP_DIRECT
8	Structural constituent of ribosome	GOTERM_MF_DIRECT
9	rRNA processing	GOTERM_BP_DIRECT
10	Cytosolic large ribosomal subunit	GOTERM_CC_DIRECT
11	Cytosolic small ribosomal subunit	GOTERM_CC_DIRECT
12	Poly(A) RNA binding	GOTERM_MF_DIRECT
13	Focal adhesion	GOTERM_CC_DIRECT
14	Membrane	GOTERM_CC_DIRECT
15	RNA binding	GOTERM_MF_DIRECT
16	Small ribosomal subunit	GOTERM_CC_DIRECT
17	Cytosol	GOTERM_CC_DIRECT
18	Intracellular ribonucleoprotein complex	GOTERM_CC_DIRECT
19	Extracellular exosome	GOTERM_CC_DIRECT
20	Extracellular matrix	GOTERM_CC_DIRECT
21	Ribosomal large subunit assembly	GOTERM_BP_DIRECT
22	Nucleolus	GOTERM_CC_DIRECT
23	Cytoplasmic translation	GOTERM_BP_DIRECT

## Data Availability

The data used to support the findings of this study have been deposited in the Gene Expression Omnibus repository (https://www.ncbi.nlm.nih.gov/geo/query/acc.cgi?acc=GSE161731).

## Abbreviations

mRMR: Max-Relevance and Min-Redundancy
IFS: Incremental feature selection
RF: Random forest;
MI: Mutual information
MCC: Matthew's correlation coefficient
DT: Decision tree
SVM: Support vector machine
kNN: *K*-nearest neighbor

RETRACTED

## Supplementary Materials

Supplementary 1 Table S1: 15937 features (genes) to represent each acute respiratory infection sample.

Supplementary 2 Table S2: mRMR feature list generated by mRMR method.

Supplementary 3 Table S3: performance of IFS with different classifiers.

Supplementary 4 Table S4: rules generated from DT analysis.
